# Influencing Factors of CO_2_ Emissions in Chinese Power Industry: A Study from the Production and Consumption Perspectives

**DOI:** 10.1155/2022/3615492

**Published:** 2022-05-04

**Authors:** Qiang Liu, Chunmei Mao, Fan Tian

**Affiliations:** ^1^School of Business, Hohai University, Nanjing 211100, China; ^2^School of Public Administration, Hohai University, Nanjing 211100, China; ^3^Lianyungang E-port Information Development Co., Ltd, Lianyungang 222042, China

## Abstract

China's huge regional differences are taken into consideration to study the influencing factors and their differences in CO_2_ emissions of the power industry from different regions. This study aimed to improve the efficiency of CO_2_ emission reduction policies. From the production and consumption perspectives, this study analyzes the influencing factors of CO_2_ emissions and utilizes the Logarithmic Mean Divisia Index (LMDI) to decompose CO_2_ emissions with consideration of the cross-regional power dispatching in the power industry. The results indicate that the trend of CO_2_ emissions in the eastern, central, and western China seems similar during years 2005 to 2017 no matter from which perspective. From the production perspective, power consumption is the main factor in CO_2_ emission increase and its affect extent may vary from different regions over a period of time. Energy efficiency inhibits CO_2_ emission increase in all regions. The power structure and power distribution across regions affect CO_2_ emissions significantly different in amount and direction from region to region. From the consumption perspective, economic activity plays a major role in CO_2_ emission increase and plays a similar role in the trend of CO_2_ emissions in three regions, but its affect extent on CO_2_ emissions varies in different regions. Targeted policy recommendations are provided to reduce CO_2_ emissions more effectively from China's power industry.

## 1. Introduction

Climate change caused by excessive carbon emissions is a serious threat to nature. China replaced the United States in 2006 to become the world's largest carbon emitter along with rapid economic development. After realizing the urgency of reducing CO_2_ emissions, the Chinese government has decided to reduce carbon intensity by between 55% and 60% [1]. In addition, China committed to peak carbon emissions by 2030 at the Asia Pacific Economic Cooperation (APEC) in 2014 [2], but it is not easy for China to fulfill this commitment [3]. The power industry in China is high in energy consumption and emission, which accounts for 50% of coal consumption and 40% of CO_2_ emissions in China [4]. Apparently, the power industry should therefore be the priority to reduce CO_2_ emissions. However, China is with regional differences in natural resources, economy, population, and technology. Taking this into account, we aimed to study the regional differences in CO_2_ emissions in the Chinese power industry in order to improve the carbon emission efficiency.

It is noteworthy that more scholars began to pay attention to the influencing factors of regional differences in CO_2_ emissions. Some scholars have analyzed carbon inequality between countries and explained the root reasons for global inequality during the sample period [5, 6]. Malla (2009) [7] discussed the factors influencing the evolution of carbon emissions from the power industry in several countries. Its results have shown that the influencing extent of factors on CO_2_ emissions varied in different countries. Except for studies among countries, some research studies have examined differences among regions in emissions within a broad country such as China. Liu et al. [8] studied GHG emission characteristics, trends, and influencing factors of four Chinese cities and concluded that emission reduction policies should vary in different cities. Chen et al. [9] studied regional differences in CO_2_ emissions generated by coal consumption and explained that the root reason for emission differences is the disparity in economic growth. Moreover, some scholars have studied interregional differences in CO_2_ emissions in the power industry. Wen and Yan [10] used a panel data model to study factors driving CO_2_ emissions from the Chinese power industry from the regional and provincial perspectives. The results have shown that the impacts were different across regions. Zhou et al. [11] assessed the multiple factor impact of CO_2_ emissions from power generation at the regional grid level from 2004 to 2010. The research found that the power grid in the northern China performed poorly. Yan et al. [12] further analyzed regional differences in power consumption and predicted CO_2_ emissions for each region from 2013 to 2020 on the basis of Zhou et al.'s [11] paper.

Nevertheless, previous research studied the regional differences and driving factors of CO_2_ emissions in the power industry only from a single perspective of production and did not consider the balance between producer responsibility and consumer responsibility in emissions, which to some extent weakens the emission reduction effect. Carbon leakage is likely to be caused when producer responsibility is employed to calculate CO2 emission of power industry which means CO2 emission from the power industry in each region is equal to direct CO2 emission from thermal power generation. This method ignores the phenomenon of carbon leakage in interprovincial power dispatching and characteristics of interregional power dispatching.

Scholars have studied regional carbon emissions from the consumption perspective due to power dispatching complexity. Wang et al. (2017) [13] extended the methods of Kang et al. (2012) [14] and Ji et al. (2016) [15] to propose a new estimation method, which is relatively accurate to measure CO_2_ emissions of regional consumer. There is vast power dispatching around China with the power grid construction to solve the contradiction of power supply and demand. Some scholars have proved that CO_2_ emissions are significantly different under different measurement perspectives. It is unilateral for either producers or consumers to undertake emission reduction obligations. The accounting scheme of carbon emission responsibility based on producers and consumers should be adopted to solve the imbalance of CO_2_ emissions in the regional power industry [16].

The paper adopts the method of Wang et al. [13], Kang et al. [14], and Ji et al. [15] to calculate regional CO_2_ from both production and consumer perspectives. The core idea of “carbon accounting” schemes is to consider the spatial transfer of emissions caused by power trading to fully reflect consumers' environmental responsibility. It is more conducive to reveal the real situation of carbon emission transfer among regions to study from both production and consumption perspectives and provide correct suggestions for carbon emission reduction. Therefore, this study employs Wang et al.'s [13] method to calculate regional CO_2_ emissions from the production and consumption perspectives.

The commonly used approach in previous papers to study the impact of factors on carbon emissions from the energy industry is the LMDI due to its adaptability, availability, and easy interpretation of results (Ang 2004) [17]. The main driving factors at present affecting CO_2_ emissions from the power industry are divided into economic and social factors (economic activities, population, etc.), structural factors (energy structure, industrial structure, etc.), and efficiency factors (energy efficiency, consumption efficiency, etc.) [4, 10, 18–20]. However, seldom scholars regard power dispatching as a factor affecting carbon emissions. With the power dispatching increase, it should be considered as an influencing factor of CO_2_ emissions caused by power generation [20]. Even if some scholars have taken power dispatching as a driving factor in carbon emission, research was studied at the national level but without taking regional differences into account. We argue that there should be differences in the impact of power dispatching on carbon emissions in power import and export regions.

The current existing literature rarely considered power dispatching as a driving factor when studying regional differences in CO_2_ emissions in the power industry. This usually leads to deviations in the accuracy of assessment results. On this basis, we first divide China into three regions based on different economic and geographic distributions and then calculate regional CO_2_ emissions from the power industry from the production and consumption perspectives, respectively. Finally, we employ the LMDI method to determine the factors influencing the regional CO_2_ emissions of China's power industry from two perspectives. Compared with existing research, we intend to contribute in two ways: (1) this study analyzes the variation trend of regional carbon emissions from both production and consumption perspectives under consideration of mass cross-regional power dispatching in China's power industry, which makes the analysis results more systematic and comprehensive. (2) Moreover, this study also divided CO_2_ emission influencing factors from the power industry into production factor and consumption factor, which can determine influencing factors on CO_2_ emissions from the regional power industry more accurately, and provided valuable suggestions for China to formulate more effective policies on carbon emission reduction.

The rest of the study is structured as follows.  Section 2 introduces the main calculation method and data description.  Section 3 presents the decomposition results and discussion.  Section 4 summarizes the paper and provides policy recommendations.

## 2. Methods and Theory

### 2.1. Production Perspective

#### 2.1.1. Estimate CO_2_ Emissions from the Production Perspective

We apply the method provided by the Intergovernmental Panel on Climate Change (IPCC) to calculate CO_2_ emissions from thermal power generation in one region from the production perspective without considering power dispatching across regions. The CO_2_ emission formula for the given region is as follows:

(1) $$\begin{array}{c} C^{a}=\sum_{i}C_{i}^{a}=\sum_{i}F_{i}\times K_{i}\times \varepsilon_{i}\times \gamma_{i}\times \frac{44}{12}, \end{array}$$

where *C*^*a*^ is the CO_2_ emission amount from burning of fossil fuels in one area. *i* is the fossil fuel type. *F*_*i*_ is the quantity of the *i*th fossil fuel in this area. K is the net heating value. *ε*_*i*_ is the oxidizer of carbon. *γ*_*i*_ is the carbon emission coefficient. 44/12  is the molecular weight ratio. We assume that the carbon emission coefficients of various fuels remain constant during the study period. Although the coefficients vary over time due to changes in fossil fuel grade, these changes are relatively small. Therefore, it can be ignored in the analysis of more important coefficients in CO_2_ emissions [18].

#### 2.1.2. Decomposition Method from the Production Perspective

Decomposition from the production perspective of CO_2_ emission is expressed as follows:

(2) $$\begin{array}{c} C^{a}=\frac{C^{a}}{E}\frac{E}{Q_{F}}\cdot \frac{Q_{F}}{Q_{P}}\cdot \frac{Q_{P}}{Q_{T}}\cdot Q_{T}, \end{array}$$

where *E* is the fossil fuel consumption for thermal power generation in the region. *Q*_*F*_ is the thermal power generation in the region. *Q*_*P*_ is the overall amount of power generated in the region (including thermal power and hydroelectric power). *Q*_*T*_ is the total power consumption in the region (including final consumption and transmission loss).

Equation (2) is equivalent as follows:

(3) $$\begin{array}{c} C^{a}=CC\cdot EE\cdot ES\cdot IO\cdot Q. \end{array}$$

The function could be edited as follows according to the LMDI additive decomposition method:

(4) $$\begin{array}{c} \Delta C^{a}=C_{t_{2}}^{a}-C_{t_{1}}^{a}=\Delta C_{CC}+\Delta C_{EE}+\Delta C_{ES}+\Delta C_{IO}+\Delta C_{Q}. \end{array}$$

According to the LMDI additive decomposition method, we decompose the overall change amount (△C) of CO_2_ emission from the power industry into five influencing factors based on the producer responsibility in the base year and target year. *CC* is the carbon emission coefficient. Δ*C*_*CC*_ is the impact of the fossil fuel structure change. *EE* is the energy efficiency of thermal power. Δ*C*_*EE*_ is the influence of the energy conversion efficiency change in thermal power. *ES* is the power structure. Δ*C*_*ES*_ is the change influence of power structure on CO_2_ emission. *IO* is the power dispatching across regions. Δ*C*_*IO*_ is the impact of changes in power distribution across regions.  *Q* is the power consumption. Δ*C*_*Q*_ is the impact of changes in power consumption on CO_2_. *t*_2_ and *t*_1_ are base year and target year, respectively (*t*_2_ > *t*_1_).

We utilize the following formulas to calculate these driving factors:

(5) $$\begin{array}{c} \Delta C_{CC}=L\left(C_{t_{2}}^{a}-C_{t_{1}}^{a}\right)\cdot \;\ln\left(\frac{CC_{t_{2}}}{CC_{t_{1}}}\right), \end{array}$$

(6) $$\begin{array}{c} \Delta C_{EE}=L\left(C_{t_{2}}^{a}-C_{t_{1}}^{a}\right)\cdot \;\ln\left(\frac{EE_{t_{2}}}{EE_{t_{1}}}\right), \end{array}$$

(7) $$\begin{array}{c} \Delta C_{ES}=L\left(C_{t_{2}}^{a}-C_{t_{1}}^{a}\right)\cdot \;\ln\left(\frac{ES_{t_{2}}}{ES_{t_{1}}}\right), \end{array}$$

(8) $$\begin{array}{c} \Delta C_{IO}=L\left(C_{t_{2}}^{a}-C_{t_{1}}^{a}\right)\cdot \;\ln\left(\frac{IO_{t_{2}}}{IO_{t_{1}}}\right), \end{array}$$

(9) $$\begin{array}{c} \Delta C_{Q}=L\left(C_{t_{2}}^{a}-C_{t_{1}}^{a}\right)\cdot \;\ln\left(\frac{Q_{t_{2}}}{Q_{t_{1}}}\right). \end{array}$$

L is the logarithmic mean value: $L\left(x,y\right)=\left\{\begin{array}{cc} y-x/\ln\;y-\ln\;x, & x\neq y\\ x, & x=y \end{array}\right.$.

### 2.2. Consumption Perspective

#### 2.2.1. Decomposing CO_2_ Emissions from Consumption Perspective

Local power consumption should be taken into account when calculating the overall CO_2_ emissions in the region. CO_2_ emissions from power utilization are estimated as follows:

(10) $$\begin{array}{c} C=C^{a}+C^{b}, \end{array}$$

where C is the actual CO_2_ emissions in the region based on consumer responsibility. *C*^*b*^ is the CO_2_ emission allocation due to cross-regional power dispatching, which will be discussed in the next section. *C*^*a* ^ is the CO_2_ emissions from thermal power in the region. *C*^*b*^ is the CO_2_ emission allocation in the region. We classify all provinces into two types according to Wang et al. (2017) [13].

(11) $$\begin{array}{c} \Delta =I-O, \end{array}$$

where Δ is the net power consumption of one province. O is the output power from one province, while I is the input power from other provinces. Δ > 0 means that the input power exceeds output power, and the province will be regarded as power import province. Δ < 0 means that the output power exceeds input power, and then, the province will be regarded as power export province. We assume that each province gives priority to power production of its own.

#### 2.2.2. Decomposing CO_2_ Emissions in Power Export Provinces

(12) $$\begin{array}{c} C_{m}^{b}=\Delta \times \frac{Q_{F_{m}}}{Q_{p_{m}}}\times \frac{C_{F_{m}}}{Q_{F_{m}}}, \end{array}$$

where *C*_*m*_^*b*^ is the power export province. *m* is CO_2_ emission dispatching. *Q*_*F*_*m*__ is the thermal power produced by province *m*. *Q*_*p*_*m*__ is the overall power produced by province *m* (including thermal power generation and hydroelectric power generation). *Q*_*F*_*m*__/*Q*_*p*_*m*__ is the ratio of the thermal power generation to total power generation in province *m*. *C*_*F*_*m*__ is the CO_2_ emissions from thermal power generation in province *m*. *C*_*F*_*m*__/*Q*_*F*_*m*__ is the emission factor of the thermal power generation.

#### 2.2.3. Decomposing CO_2_ Emissions in Power Import Provinces

(13) $$\begin{array}{c} C_{n}^{b}=\Delta \times \frac{\sum_{m=1}^{m}\left|C_{m}^{b}\right|}{\sum_{m=1}^{m}Q_{F_{m}}}\times \frac{\sum_{m=1}^{m}Q_{F_{m}}}{\sum_{m=1}^{m}Q_{T_{m}}}, \end{array}$$

where *C*_*n*_^*b*^ is the dispatch of CO_2_ emissions in the power import province.

∑_*m*=1_^*m*^|*C*_*m*_^*b*^|/∑_*m*=1_^*m*^*Q*_*F*_*m*__ is the power emission factor of the total output thermal power generation, and *Q*_*F*_*m*__ is the thermal power generation distributed from province *m*.

∑_*m*=1_^*m*^*Q*_*F*_*m*__/∑_*m*=1_^*m*^*Q*_*T*_*m*__ is the ratio of dispatching amount on thermal power generation to total power dispatching. *Q*_*T*_*m*__ is the total export power of the power output province (including thermal power generation and hydroelectric power generation).

#### 2.2.4. Decomposition Method from the Consumption Perspective

According to Kaya (1989) [21] and considering the importance of industrial structure change, we decompose the exponent of CO_2_ emissions from consumption perspective as follows:

(14) $$\begin{array}{c} C=\frac{C}{Q_{T}}\cdot \frac{Q_{T}}{\text{GDP}}\cdot \frac{\text{GDP}}{P}\cdot P. \end{array}$$

Its abbreviation is as follows:

(15) $$\begin{array}{c} C=CI\cdot EI\cdot EA\cdot P. \end{array}$$

GDP is the gross domestic product of the region. P is the resident population of the region. Similar to the above description, the annual rate of CO_2_ increase can be decomposed into the following formula:

(16) $$\begin{array}{c} \Delta C=C_{t_{2}}-C_{t_{1}}=\Delta C_{CI}+\Delta C_{EI}+\Delta C_{EA}+\Delta C_{P}, \end{array}$$

where *CI* is the carbon intensity of power consumption, reflecting the cleanliness of power consumption in the region. Δ*C*_*CI*_ is the influence of power consumption on carbon intensity changes. *EI* is the power intensity, which reflects the industrial structure. Δ*C*_*EI*_ is the impact of power intensity changes. *EA* is the economic activities. Δ*C*_*EA*_ is the impact of economic development and change. Δ*C*_*P*_ is the impact of population size fluctuations.

The right side of (15) can be computed as equations (5)–(9), which are not listed here due to limited space.

### 2.3. Data Description

Considering the data accessibility and the impacts of COVID-19 pandemic on energy consumption in 2020, the Chinese power industry data from 2005 to 2019 were used in this study. We employ data on energy consumption caused by power generation in different provinces from the China Energy Statistical Yearbook (2005–2019). Besides, population data and GDP data came from China Statistical Yearbook (2005–2019). Regional GDP from 2005 to 2019 was converted on the basis of the price level in 2005. The IPCC effective CO_2_ emission factor and net calorific value of fuel were also considered. According to the geographical distribution and economic level, 30 provinces in China (Tibet, Taiwan, and Hong Kong were excluded) were divided into three parts. The detailed classification is listed in Table 1.

## 3. Results and Discussion

### 3.1. Outline of CO_2_ Emissions from the Power Industry

As shown in Figure 1, the CO_2_ emissions in three regions from 2005 to 2017 mainly go through two phases, and their trends are also similar no matter from which perspective. The first phase is from years 2005 to 2011, and the CO_2_ emissions in all regions increased significantly over time. The second phase is after 2011, and CO_2_ emissions in each region are only slightly increased and even decreased in some years. The trend of CO_2_ emissions in recent years proves that the Chinese green and low-carbon policies in the power industry have been effectively implemented. Although the overall trend of CO_2_ emissions in three regions is almost the same, it is obvious that CO_2_ emissions look higher from the consumption perspective than those from the production perspective in all tress regions.

The growth rate of CO_2_ emissions in central China was lower than the other two regions from the production perspective. The CO_2_ emissions in western China exceeded the central China from 2010 to 2011. This is mainly due to two main reasons: economic development is positively correlated with power consumption, so the developed eastern China requires a large amount of power to support its high economy. On the other hand, the economic development of western China is mainly extensive and it has carried on enterprise with high CO_2_ emissions from other regions during industrial development and upgrading of China's industries.

The growth rate of CO_2_ emissions in the eastern China was apparently the highest from consumption perspective. The current economic development needs power support, and the high economic aggregate in eastern China is precisely supported by large quantities of power consumption. This will become even more evident under the principle of “People who consume who take the responsibility.” In general, the eastern China is with the highest carbon emissions from either production perspective or consumption perspective. Therefore, the eastern China should play a leading role in carbon reduction projects in the power industry. In addition, Figures 1(a) and 1(b) indicate that the regional amount and growth rate of CO_2_ emissions are significantly different and the consumption side is higher than the production side in three regions from both perspectives.

Therefore, the analysis from two perspectives can provide a more systematic and comprehensive understanding of regional differences in CO_2_ emissions in the power industry.

### 3.2. Results and Discussion from the Production Perspective

We discuss the impact of driving factors of three regions on CO_2_ emissions from the Chinese power industry in this section. The power consumption is the most important factor for CO_2_ generation in all regions, which is known from results (as shown in Figure 2 and Table 2). The energy efficiency is the major factor in restraining every region's CO_2_ emissions even though the energy efficiency improvements in the west were not significant at the beginning of the study. The power generation structure and cross-regional power distribution have different effects on CO_2_ emissions in terms of scale and direction in three regions. The carbon emission coefficient is not the main driving factor compared with other factors during the study period. We will discuss more details in the following parts.

#### 3.2.1. Carbon Emission Coefficient and Energy Efficiency

Changes in carbon emission coefficient have a relatively low impact on CO_2_ emissions compared with other factors in all regions. It reflects that the change in fossil fuel structure in the thermal power generation is small. The ratio of coal in total fossil fuel for the thermal power generation has always remained above 90% and has no signs of decline as shown in Table 3. Generally speaking, the fossil energy structure mainly depends on the overall regional resources. In China, the structure of fossil energy has been in a state of “more coal, less oil, and shortage of natural gas.” The raw coal occupies 70% of energy consumption and will not change greatly in a short time [16]. The results show that the changes in fossil fuel structure affecting CO_2_ emissions in the power industry are weak. It also proves that there is still a long way to change the mix of fossil fuels in the thermal power generation in all regions.

The energy efficiency of thermal power generation is the main factor to restrain CO_2_ emissions from the power industry in all regions. The CO_2_ emission reductions in the eastern, central, and western China reached 43.25%, 39.86%, and 21.05%, respectively (Table 2). Although energy efficiency increased in all regions from 2005 to 2019, it had a smaller impact on CO_2_ emission reduction in the western China than in the rest of the two regions. Additionally, we can see from Table 4 that the initial energy efficiency level is inconsistent in three regions during the study period and decreased from the east to the west. These phenomena are mainly caused by two reasons: (1) the economy of the central and western regions is relatively backward, which still keeps following the traditional extensive growth model. Both the central China and western China pay little attention to environmental protection; (2) it is also directly related to the resource they owned. For example, the environmental cost of hydro-rich provinces such as Sichuan and Yunnan is lower than the cost of coal-fired power. As a result, the production capacity of thermal power in these regions is not fully utilized and the energy efficiency of thermal power generation is low. Based on differences in energy efficiency in regions, the central China and western China have great potential to improve technologies of energy conversion.

#### 3.2.2. Power Generation Structure and Cross-Regional Power Consumption

Hydropower is taken as the main comparison of power generation structure change. The power generation structure influences CO_2_ emissions in three regions varied in scale and direction. The total CO_2_ emission changes in the eastern, central, and western China are 3.09%, 3.79%, and -18.79%, respectively. As Figure 2 demonstrates, power generation structure changes slightly influence CO_2_ emissions in eastern China, while greatly influencing fluctuations of CO_2_ emissions in central China and greatly restraining CO_2_ emissions in western China. These differences are mainly caused by uneven resource distributions in regions. There is around 70% of hydroelectric power generated from western China from a national perspective. However, it is 40% of hydroelectric power generated from the west and less than 10% of hydroelectric power generated from the east from a regional perspective (Figure 3). Although the eastern China takes a low ratio in hydropower generation, it has little potential to increase this proportion (from technology perspective). The exploitable hydropower in the east coast of China only accounts for about 6% of the total power supply, while the exploitable power in the southwest, northwest, south, and central China accounts for 92%. Hence, by the end of March 2021, there is no room for hydropower exploitation on the east coast of China, compared with more than 50% exploitable space in the western China [22]. Therefore, China should focus on optimizing the energy structure of power generation in the central and western China, especially in the western China, which is rich in natural resources. Power generation structure improvement is an efficient measure to reduce emissions, which can not only ensure the power generation but also avoid environmental pollution.

The unbalanced distribution of regional natural resources is also one of the reasons affecting power dispatching. China has begun to implement power distribution measures since the 1990s to solve the mismatch problem of regional power supply and demand. Figure 2 illustrates that the impact on scale and direction of power distribution on CO_2_ emissions is inconsistent among regions. The power dispatching increases CO_2_ emission in eastern and central China while promoting the CO_2_ emissions in western China.

Although power dispatching plays different roles in different regions, it is beneficial to restrain CO_2_ emissions from the power industry. Thus, increased efforts will continue to make power dispatching. The suppression effect on CO_2_ emission of power transfer in eastern China is mainly because power import can not only solve the problem of insufficient power supply but also has a relatively low cost compared with power generation technology improvement. Therefore, the ratio of power imports is increasing year by year.

The effect of power dispatching on CO_2_ emissions in western China is by promoting to suppress, and it is because the western China has already transferred natural resource advantage into economic advantage through power dispatching. With hydropower ratio growth, the western China benefits from providing clean energy to the east and reduces local environmental pollution as well [23, 24]. In addition, the import power of central China declines, indicating that power generation pressure in the central China has shifted in search of lower economic costs. China will continue to vigorously promote power dispatching to address the imbalance between supply and demand and reduce emissions by current policies. Thus, western China should accelerate the improvement of energy efficiency and power generation structure with increased power dispatching.

#### 3.2.3. Power Consumption

Power consumption is the primary factor that increases CO_2_ emissions of the power industry with an impact of 158.39%, 170.12%, and 147.91% on overall CO_2_ emissions in eastern, central, and western China, respectively. According to Figure 2, the impact of power consumption on CO_2_ emissions from the power industry is almost consistent with the economic cycle. Mi and Zhao (2012) [25] have verified the Granger causality between power consumption and economic development. They believe that economic development inevitably leads to power consumption, and power consumption will support economic development in turn. It is interesting to find out that although three regions are different in initial economic levels, the power consumption has almost the same tendency to affect CO_2_ emissions from the power consumption. As a result, we could not simply assume that the CO_2_ emission growth rate caused by power consumption is lower in central and western China because of the lower level of economic development.

Moreover, Figure 2 indicates that the enhancement effects of power consumption on CO_2_ emissions in the power industry reduce in all regions since 2011, especially in the central China. Nevertheless, the power consumption restriction has its limitation in reducing CO_2_ emissions due to tons of power required in regional development. High economic development and intensive population in eastern China lead to high power consumption demand. The acceleration of industrialization also required huge amounts of power in western China. Compared with western and eastern China, the central China is a transitional zone and its power consumption has a relatively lower impact on CO_2_ emissions, but its power consumption, which remains stable, has no trend of decline.

### 3.3. Results and Discussion from Consumption Perspective

Economic activity is the main factor leading to CO_2_ emission increase in three regions, and affecting trends in all regions seem similar, but CO_2_ emissions in 2017 from economic activity in eastern China increased rapidly. Still, the carbon intensity and power intensity of power consumption are two key factors to restrain CO_2_ emissions and these two factors influence CO_2_ emissions, which vary from region to region. The population density has a relatively lower effect compared with other drivers.

#### 3.3.1. Carbon Intensity of Power Consumption

The carbon intensity of power consumption is an intensity index to measure the cleanliness of regional power consumption from the consumption perspective. It plays a positive role in reducing CO_2_ emissions, which accounts for -46.82%, -46.19%, and -61.83% of overall CO_2_ emission changes in eastern, central, and western China, respectively, during the study period (Table 5). Contrary to the above energy efficiency factors, the carbon intensity of power consumption in western China is the lowest, indicating that power consumption in western China has the highest cleanliness (Table 6).

The western China has no responsibility to bear CO_2_ emissions generated by power output, and its carbon intensity of power consumption can accurately measure the power consumption cleanliness. However, the power consumption cleanliness in western China decreased in 2017, which might be affected by extensive industry migration. Besides, the clean energy development in central and western China is also an important reason for the highest cleanliness of power consumption in the western China. As Figure 4 demonstrates, the carbon intensity of power consumption has a low impact on CO_2_ emissions in three regions at the beginning of the study while increases significantly in the later stage, which is mainly attributed to the cleanliness improvement of power consumption due to the rapid growth of hydropower in the central and western China at the end of the study. The power consumption cleanliness improves greatly and plays a role in restraining CO_2_ emissions in the eastern China due to the implementation of power transmission project. The carbon intensity of power consumption is an index influenced by multiple factors, including the cleanliness of region that only produced power and imported power. Everyone should work together to improve the power consumption cleanliness.

#### 3.3.2. Power Intensity

Power intensity represents the dependence of GDP on power consumption. Its change reflects the influence of industry structure change. Although the power intensity promotes the CO_2_ emissions in western China during the study period, it is the main factor in reducing CO_2_ emissions in all regions. Compared with eastern and central China, the change in power intensity in western China has less impact on CO_2_ emissions. This is mainly due to different industrialization levels in three regions.  Table 7 demonstrates that there are significant differences in power intensity levels of three regions. The power intensity decreases progressively from east to west, which reflects the differences in the original industry structure among regions. The greater the dependence of GDP on power consumption, the greater the ratio of secondary industry in the region.

After a series of national strategies issued, some high-consumption and high-polluting industries have been moved inland and the overall economic growth disparities among regions have been gradually reduced [26, 27]. The results indicate that the reduction in secondary power consumption in western China is not obvious, but the industry structure has gradually improved in the western China. Actually, the Chinese government acknowledges that the industry transfer can only eliminate regional economic differences, but not reduce total CO_2_ emissions. Thus, the backward heavy industry technologies and industries in all regions should be eliminated to reduce total carbon emissions.

#### 3.3.3. Economic Activity

The per capita GDP is a comprehensive indicator reflecting economic growth and quality of life. Figure 4 indicates that economic activity is the first driving factor for CO_2_ emission increase from the power industry in all regions. The overall change in three regions increased by 177.50%, 209.06%, and 178.44%, respectively. This finding is in line with the results of Yang and Lin (2016) [4] and Zhang et al. (2013) [18]. The power generation, which is an essential element of productive activity, supports economic development. The economic development in turn gives rise to power demand and CO_2_ emission increase. There are obvious economic level differences among regions in China since the reform and opening-up [28]. However, the influences of economic activity on driving CO_2_ emissions in the three regions are in the same manner and fluctuate with the economic cycle. This is because economic activity (GDP/P) changes with the economy when the fluctuation of population scope in a region is very small. With the Chinese economy entering the new normal, the GDP growth has been transformed from rapid growth into medium-high-level growth since 2013. The economic activity makes a lower contribution to decreasing CO_2_ emissions with the development of high-quality economy.

Scholars have proved that economic growth and environmental pollution have an inverted U-shaped relationship. There is still a long way for eastern China to reach the inflection point of inverted U shape of the most economically developed region in China. Thus, the economic activity will become the major driving factor in environmental pollution for a long time [29, 30], but economic activity can restrain CO_2_ emissions from the power industry to some extent. For instance, officials in prosperous regions have a strong sense of environmental protection, while officials in impoverished regions are limited to economic development. Therefore, maintaining high-quality economic development is an effective way to slow down CO_2_ emissions.

#### 3.3.4. Population Size

The impact of population size on CO_2_ emissions can be ignored compared with other influencing factors. The change in population size influences CO_2_ emissions more obvious in eastern China compared with the rest of the two regions. The eastern China has a large population, which is mainly because of massive influx of people attracted by its blossom. Overall, population size has little effect in CO_2_ emissions and it will not change much in the coming years [19].

## 4. Conclusions

This study aims to study regional differences in CO_2_ emissions from China's power industry. Due to the universality of cross-regional power dispatching in the power industry, different regions have different CO_2_ emission responsibility from the production and consumption perspectives. This study decomposes CO_2_ emissions by LMDI and determines the factors affecting CO_2_ emissions from both mentioned perspectives. Based on the decomposition results from 2005 to 2017, we observe significant differences in factors influencing CO_2_ emissions from the power industry in scale and direction among regions. Therefore, measures to reduce CO_2_ emissions from the power industry should vary from region to region.

This research has mainly discussed the impact of energy supply and demand distribution on carbon emissions from perspectives of energy supply and demand and power dispatching, and we aim to provide a reference for planning decision-makers and institution makers.

From the production perspective,

1. Although power consumption has a decreased influence on CO_2_ emissions in recent years, it remains the leading factor increasing CO_2_ emissions in all regions. It is unrealistic in practice to control CO_2_ emissions by restraining power consumption, especially in the eastern and western China. However, the Chinese government can enforce economic regulations to avoid excessive demand, which will contribute to reducing CO_2_ emissions.
2. Energy efficiency is the main factor restraining CO_2_ emissions in all regions, but the initial levels of energy efficiency in different regions are significantly different. The central China and western China still have plenty of room to improve energy efficiency compared with the eastern China. Thus, the government should increase financial investment in energy efficiency in these two regions, such as continuing to restrict small-scale power generation enterprises and encouraging advanced energy conversion technologies.
3. In addition, power structure and power distribution affect CO_2_ emissions differently in scale and direction in three regions. Therefore, measures to reduce CO_2_ emissions should vary from region to region. For example, the central and western China should take advantage of rich resources to optimize the power generation and thus reduce carbon emissions. Moreover, the eastern China should increase the dispatching of project to send power from the west to the east with the increase in hydroelectric power generation, so that the eastern China can fully benefit from hydropower of other regions.

From the consumption perspective,

1. Economic activity is the major factor to increase CO_2_ emissions in all regions, and its influences on increasing CO_2_ emissions in all regions bear out the similar trend. As the economy grows, the local government should increase fiscal spending on environmental protection, especially in less developed areas where officials lack adequate awareness of environmental protection. In addition, China should always pay attention to the economic growth quality and accelerate the transformation of economic model from extensive to intensive.
2. The power intensity should keep improving despite that the overall CO_2_ emissions continue to rise. The carbon intensity of power consumption and power intensity are main restraining factors to CO_2_ emissions in all regions, and their influences vary in different regions. It is wisdom for the Chinese government to implement industry transformation policies given that different regions are different in industrialization and economic development. The eastern China has transferred energy-intensive and heavily polluting industries to the central and western China as they have abundant natural resources and favorable markets, which can reduce the energy loss and cost during transportation.

However, the regions that industry moves into should reject the backward industries to avoid carbon leakage and achieve the overall goal of low CO_2_ emissions. To sum up, reducing CO_2_ emissions is not a simple unilateral action. The Chinese government should recognize regional differences and adopt targeted policies from the production and consumption perspectives to create a “low-carbon environment” for the power industry.

From the perspective of cross-region power dispatching policy:

(1) This study discussed the cross-region power allocation, which was viewed as an effective energy-carbon allocation measure. Currently, from the perspective of practice, the effectiveness of this allocation measure is mainly reflected in two aspects: (1) the cross-region power dispatching is in accord with the reality that the energy distribution does not match with the population and industry distribution in China. The energy supply in China is mostly located in the western region, while the major electricity demand from production and life is located in the coastal economic belt. Without long-distance power dispatching, most renewable energy could not be totally consumed by the local region. (2) In China, most of the renewable energy supply comes from underdeveloped regions, which have low payment capacity for energy consumption. The cross-region power dispatching could effectively improve the economy of renewable energy from the demand side, which would contribute to the carbon emission reduction process in China. This effectiveness could be viewed as the imbalance consideration of natural distribution on the supply and demand side in regional energy planning. Hence, cross-region power dispatching is generally an irresistible choice, which is similar in developed regions such as Europe and the United States. In fact, although the new petrochemical power company in the western China would generate large carbon emissions, the cross-regional scheduling is beneficial due to the advanced energy efficiency and its contribution to the stability of the power system. This is also an episode in the process of technological change in the power industry.

### 4.1. Based on This, We Further Discuss Two Issues

When will this trans-regional power dispatching be ineffective? Apparently, it will result in an overall carbon emission increase to relocate power supply utilities from developed regions to underdeveloped regions simply because of carbon regulation. Moreover, the trans-regional power dispatching might result in comparative advantages of carbon permit only because of the difference in development among regions. To be specific, the carbon price is low in central and western regions thanks to abundant carbon sinks, while traditional power generation enterprises move westward because of the shortage of carbon permit. In this vein, trans-regional power dispatching should be assessed whether the increase in the economic development of western underdeveloped regions by this dispatching is worth the carbon emission generated by it. In the context of global carbon neutrality, this comparative advantage will disappear with the improvement of the balanced regional development and the diffusion of low-carbon technologies. As a result, the extent of trans-regional power dispatching will be suppressed.

Under what circumstances would this trans-regional power dispatching be more effective? In addition to the trans-regional power dispatching driven by high demand, the difference in the development intensity and potential of renewable energy among different regions are the natural driving factors for trans-regional power dispatching. From the perspective of supply side, preferential access, preferential dispatching, and preferential pricing of low-carbon power are the institutional motivation of trans-regional dispatching. From the demand side, the pricing system of integrated energy price, which includes carbon price, trading system of power system, and subsidy system of low-carbon electricity, will make it more feasible and efficient to promote trans-regional power dispatching of renewable energy power. Generally speaking, pricing market transactions and priorities of supply and demand can not only directly affect the supply and demand relationship of low-carbon power but also affect the possibility and utility of trans-regional power dispatching of low-carbon power.

Finally, we try to discuss the similarities and differences between China and Europe in power dispatching and relevant policies. Since the operation of ENTSO-E in 2009, the EU has established a unified power market in the form of an operator alliance, and the proportion of transnational exchange electricity is about 15%. In particular, typical countries include Denmark (dominated by thermal and wind power), Norway (dominated by hydropower), and Sweden (dominated by hydropower and nuclear power). Due to the differences in energy distribution and demand, electricity exchange between countries is common. The unified grid connection and standard would be valuable for Europe, and a flexible electricity price system and even negative electricity price (encouraging users to use off-peak electricity) and accurate power accounting ability in Europe would be valuable for China. Besides, studies in Europe show that carbon tax, carbon price, and the improvement of cross-border transmission capacity could contribute to the production of low-carbon electricity [31, 32].

## Figures and Tables

**Figure 1:** CO_2_ emissions from the power industry in three regions from 2005 to 2017: (a) CO_2_ emissions in three regions from the production perspective. (b) CO_2_ emissions in three regions from the consumption perspective.

**Figure 2:** Contribution value of different factors on CO_2_ emissions in three regions from the production perspective: (a) eastern China, (b) central China, and (c) western China.

**Figure 3:** Hydropower generation ratio: (a) regional hydropower generation ratio in China and (b) hydropower generation ratio in overall power generation.

**Figure 4:** Contribution of different drives to CO_2_ emissions in three regions from the consumption perspective: (a) eastern China, (b) central China, and (c) western China.

**Table 1:** Detailed classification of the Chinese regional divisions.

Regions	Provinces
East regions	Beijing, Tianjin, Hebei, Liaoning, Shanghai, Jiangsu, Zhejiang, Fujian, Shandong, Guangdong, Hainan
Central regions	Shanxi, Jilin, Heilongjiang, Anhui, Jiangxi, Henan, Hubei, Hunan
West regions	Chongqing, Sichuan, Guizhou, Yunnan, Shaanxi, Gansu, Ningxia, Qinghai, Xinjiang, Guangxi, Inner Mongolia

**Table 2:** Changes in overall CO_2_ emissions by different factors from the production perspective from 2005 to 2019 (unit: in metric tons).

Effect	Eastern China	Percent	Central China	Percent	Western China	Percent
△CC fuel structure	143.54	17.03%	29.52	6.02%	6.73	0.85%
△EE energy efficiency	−364.51	−43.25%	−195.32	−39.86%	−166.94	−21.05%
△ES electricity structure	26.04	3.09%	18.57	3.79%	−149.06	−18.79%
△IO interregional power dispatching	−320.89	−38.08%	−123.83	−25.27%	35.21	4.44%
△Q power consumption	1358.57	161.21%	761.03	155.32%	1067.27	134.55%

**Table 3:** Ratio of raw coal in total fossil fuel consumption of the thermal power generation (unit: percentage).

Region	2005 (%)	2006 (%)	2007 (%)	2008 (%)	2009 (%)	2010 (%)	2011 (%)	2012 (%)	2013 (%)	2014 (%)	2015 (%)	2016 (%)	2017 (%)	2018 (%)	2019 (%)
Eastern region	93	94	94	94	94	95	95	94	95	94	94	93	94	94	93
Central region	97	96	96	95	95	92	93	94	93	94	93	92	93	92	92
Western region	97	98	98	97	97	97	95	95	95	95	95	93	94	94	93

**Table 4:** Energy efficiency of thermal power generation (unit: kJ/104 kW h).

Region	2005	2006	2007	2008	2009	2010	2011	2012	2013	2014	2015	2016	2017	2018	2019
Eastern region	10.22	9.75	9.42	9.38	9.14	9.03	9.14	8.9	8.68	8.47	8.17	8.3	8.07	8.21	8.17
Central region	11.6	11.45	10.89	10.98	10.46	10.42	10.42	10.19	9.75	9.64	9.35	9.27	9.33	9.31	9.58
Western region	12.12	12.11	11.7	11.91	11.49	11.11	11.47	11.21	10.42	10.16	9.91	9.79	10.2	9.83	10.06

**Table 5:** Changes in CO_2_ emission caused by drivers from the consumption perspective during 2005–2019 (unit: tons).

Effect	Eastern region	Percent	Central region	Percent	Western region	Percent
△CI	−512.7	−46.82%	−213.51	−46.19%	−314.76	−61.83%
△EI	−565.37	−51.63%	−325.69	−70.46%	−122.35	−24.03%
△EA	1943.71	177.50%	966.34	209.06%	908.42	178.44%
△P	229.42	20.95%	35.08	7.59%	37.78	7.42%

**Table 6:** Carbon intensity of power consumption (unit: *T*/102 kW h).

Region	2005	2006	2007	2008	2009	2010	2011	2012	2013	2014	2015	2016	2017	2018	2019
Eastern region	0.092	0.091	0.089	0.088	0.086	0.084	0.086	0.082	0.081	0.076	0.073	0.072	0.071	0.074	0.070
Central region	0.093	0.094	0.091	0.087	0.083	0.084	0.085	0.082	0.079	0.076	0.073	0.071	0.072	0.073	0.072
Western region	0.080	0.085	0.083	0.077	0.076	0.070	0.072	0.065	0.064	0.058	0.055	0.054	0.054	0.055	0.053

**Table 7:** Power intensity of the three regions (units: kW·h/yuan).

Region	2005	2006	2007	2008	2009	2010	2011	2012	2013	2014	2015	2016	2017	2018	2019
Eastern region	0.117	0.117	0.116	0.110	0.106	0.107	0.107	0.102	0.100	0.096	0.093	0.092	0.088	0.087	0.089
Central region	0.123	0.122	0.126	0.121	0.115	0.114	0.114	0.109	0.104	0.098	0.092	0.089	0.086	0.086	0.087
Western region	0.160	0.164	0.167	0.157	0.150	0.153	0.161	0.155	0.152	0.152	0.142	0.137	0.138	0.139	0.139

## Data Availability

The data used to support the findings of this study are included within the article. The original details of the data presented in this study are available on request from the corresponding author.
